The article "Analysis of Rational Drug Use Effect under Hospital Drug Control System" was published in 2022. Journal: Comput Math Methods Med.

# Analysis of Rational Drug Use Effect under Hospital Drug Control System

**DOI:** 10.1155/2022/2927606

**Published:** 2022-08-17

**Authors:** Haoli Huo, Xiaoyan Li, Hui Li, Haiye Wang, Xin Ma, Chen Chen, Hongfeng Zhang

**Affiliations:** Department of Pharmacy, Handan Central Hospital, Handan 056008, China

## Abstract

**Objective:**

To describe and assess the hospital drug control system's measures.

**Methods:**

From 2017 to 2019, examine the changes in medication percentage, important monitoring drug amount, top 10 medications amount, and usage rate of prophylactic antibiotics for type I incisions.

**Results:**

The proportion of pharmaceuticals remains below 30%, the number of significant monitoring drugs has decreased, the top ten drugs have shifted from adjuvant to therapeutic drugs, and the use of prophylactic antibiotics for type I incisions has decreased by 10%.

**Conclusion:**

The percentage of medications that met requirements by using the drug control system has steadily decreased, and the number of pharmaceuticals for important monitoring pharmaceuticals has steadily decreased, in accordance with national medical insurance policy, as well as improved rational drug usage.

## 1. Introduction

The State Council issued No. 38 in 2015, stating that the public hospital revenue system needed to be changed and that strict control of pharmaceutical costs was unjustified, resulting in a drop in the percentage of public hospital drugs in the pilot city (excluding Chinese medicine drinkers) to around 30% by 2017. Medication ratio management was used as a management measure by a number of medical organizations [1]. The Handan City Health and Family Planning Commission published a notice on boosting the follow-up monitoring of essential pharmaceuticals in public hospitals as the doctor's change advanced, and key medication surveillance was launched at our hospital [2]. Furthermore, the antimicrobial prophylaxis usage rate for class I incisional surgery should be less than or equal to 30%, and such medical records should be carefully verified regularly. Monthly, the quantity and amount of antimicrobial medicine usage were double sorted, and medical record spot checks were undertaken by the top 10 departments and people [3]. Every year, the top 10 medications by medication quantity were statistically analyzed and evaluated [4]. As a public tertiary general hospital at the crossroads of three provinces, our hospital bears the burden of diagnosing and treating critically ill patients in the periphery, the proportion of controlled drugs is somewhat difficult, and it may achieve certain success only by taking multiple measures, combined with clinical, pharmaceutical, and administrative interventions [5]. This study investigates the changes in drug percentage, the amount of attention paid to medication monitoring, the rate of usage of class I incision antibiotic prophylaxis, and other management indicators under various drug administration techniques in relation to the existing policy form [6].

## 2. Materials and Methods

### 2.1. Data Collection

The hospital's his system, amygdalin software, the Mecon system, relevant departmental records, and website announcements were used to collect data for this study.

### 2.2. Research Method

Statistics for 2017-2019, the percentage of total hospital medicines is monthly data, with a focus on monitoring the number of medications in the catalog used annually, the number of the top 10 drugs, and antimicrobial drug consumption in class I incision prevention. EXCAL tables were used for descriptive statistical analysis to compare changes before and after control and indicators.

### 2.3. Specific Measures

#### 2.3.1. Drug Proportion Control System

Set up a working leadership committee for the proportion of control drugs, with the dean serving as the leader and the vice dean serving as the vice leader. This will improve medicine, encourage the prudent use of clinical drugs and antibacterial treatments, reduce the drug ratio, and collaborate with our hospital. The group's office is known as the “drug control office.” The head of the drug department's clinical department is in charge of management. The leading group established a medical department, a pharmacy department, and an advocacy department to promote drug-related laws and regulations, hospital drug control-related rules and regulations, management methods, and medical modification; to raise awareness of reasonable, legal, and compliant drug use among health care workers, and to promote publicity, inspections, punishments, and rewards. Cardiovascular medications, nervous system drugs, anticancer drugs, adjuvant pharmaceuticals, and certain Chinese medicine injections lose their most critical control, and their most important monitoring is reduced in half. The Drug Control Office gathered clinical pharmacists and other clinical professionals to assess the top 20 most-prescribed medications each month. When there was a trend of super-routine or needless prescriptions, the medicine was halted for three months. For clinical departments to determine the Department drug occupancy goal, the drug control office looks at the actual to target ratio. If the decline is greater than 30%, the department bonus and director are not penalised. If the drop is less than 30%, 50% of the manager's bonus are withdrawn. For nutritional support class auxiliary medication of the hospital's key control and halving shopper medicine newly communicated by the hospital each month, the department level should strengthen the regulation, reduce the medication under the premise of reasonable drug use, and have conversations and penalties with the super routine drug use and personal record inspection departments. You cannot take part in the yearly evaluation if you use four or more drugs. Top 10 physicians with the most monthly prescription expenses were scrutinized for excessive drug usage. The doctor with the highest points for inappropriate drug usage earned an appointment, and the top doctor got a Codonopsis action each month. When the hospital's medication ratio did not achieve the overall aim, the professional or department that did not met the goal was based on their professional characteristics (the same drug ratio target professional, the standard department is not within the sequence). The doctor with the lowest average patient cost had his medical record modified to utilize POA. The doctor and department director who present with inappropriate medication administration make an appointment, minus the doctor's bonus for the month. Half of the department directors complete target management award; medical record points occur within half a year 3 unreasonable doctors to schedule an appointment, suspend prescription rights for 3 months, report to the medical department, and report to the department director by the record review department. The drug control office organizes the clinical pharmacists and other clinical experts in the department of pharmacy every month, and physicians in the top ten of time average costs, the first two of each specialty, and the first ten of class I incision surgery prevention randomly pick medical records for review. The point review department avoids. Each clinical department head is on the expert panel and must examine reasonable medication usage. Each week, the medical, pharmacy, sensory control, critical care, and laboratory medicine departments ran the rational drug use ward. Walk into a clinical department weekly, evaluate the running medical record for acceptable medication usage, and observe hospital patients. Inquire about the progress of the disease and focus on the use of antibacterial medicines, the rate of perioperative antimicrobial prophylaxis in surgical departments, the rate of antimicrobial drugs before treatment, the intensity of antimicrobial drug consumption, and the incidence of bacterial resistance. The five department union highlights pharmaceutical concerns and reacts in the department face-to-face with the clinical department.

#### 2.3.2. Antimicrobial Drug Management System

In the implementing regulations of review criteria of Hebei tertiary general hospital (2013 Edition), the operation of class I incision (2 h of surgical time) and the usage of preventive antimicrobials required to be 30 percent. In our facility, the indicator is about 55%, which is substantially more than necessary. Inguinal hernia repair (including patch repair), thyroid disease surgery, breast disease surgery, arthroscopy surgery, carotid endarterectomy, cranial mass resection, and diagnostic surgery via vascular intervention are not prophylactic for antimicrobials, according to 2015 guidelines for the clinical use of implants for the seven diseases. Antimicrobial prophylaxis in the perioperative phase should be 0.5 to 1 hour before surgery, and in class I incision surgery, it should not be more than 24 hours. Antimicrobial agents and postoperative prophylactic medicine should also be regulated. In this management, the medical record of class I incisions was obtained monthly, and the top 10 physicians rated the average prescription cost of antibacterial medicines for class I incision surgery prevention. The medical records of the doctors who ranked first for the subtotal average cost of antimicrobial prophylaxis for class I incision surgery were reviewed using point review and random spot checks. The doctors who showed unreasonable drug use were interviewed by the record review department and had their bonuses taken away for the month. The physicians with three inappropriate drug usage were also interrogated and lost their incentives. Every month, antimicrobial usage was rated. Antimicrobial medications in the top 10 total medication quantity were totalled, and the department of pharmacy created medication points. Using Mecon, medical records were abstracted and named. Medical records were also retrieved at random, with a reference to our hospital's appraisal standards for the sensible use of antimicrobial medications. Based on the grading criteria, persons or departments with fewer than 80 points were interrogated.

#### 2.3.3. Effect of Drug Management System

Handan City put out a warning to increase important medication tracking and monitoring in public hospitals. Our hospital has created clear guidelines for essential monitored pharmaceuticals and set up a working committee to handle monitoring drugs. Head of the clinical department oversees medication management. To enhance special point evaluation, monthly sales, and ranking of pharmaceuticals on the list, the doctor who initially monitored drug dose was picked at random. (In the Wellcome system, input the name of the first physician whose dose was recorded, and the medication name, i.e., medical record and prescription, was picked at random.) Before picking a medicine, physicians should weigh its benefits and costs. Also, they should respect the medicine's specifications and Medicare drug list restrictions. Doctors should not allow patients utilize medications unapproved methods. The review study focuses on prescribing medications clinically (drug selection, drug indication, use and dosage, route of administration, drug interactions, compatibility contraindications, etc.). Orders Menu included Review antimicrobial drugs, Assessment criteria for antimicrobial medication usage our hospital created, Monthly drug sequencing and review findings, an unreasonable medication caution by a doctor, and three unnecessary medical visits in half a year.

## 3. Results

### 3.1. Changes in Drug Occupancy Indexes

After developing the drug accounting control system in October 2017, clinical departments cooperated to better execute rules and regulations and reduce the drug accounting ratio while enhancing rational drug usage.  Figure 1 shows the change in medication percentages from 2017 to 2019. The drug occupancy ratio was around 41% before October 2017 and dropped to less than 30% by December. Each month in 2018 was below 30%, with late 2019 above 30%. The average drug percentage statistics for 2017 (39%), 2018 (29%), and 2019 (30%) meets national criteria.

### 3.2. Use of Antimicrobial Agents for Class I Incision Prophylaxis

In 2017-2019, the rate of class I incision prevention using antimicrobial medications was derived by our hospital's amygdalin software, as shown in Figure 2. From January to September 2017, the usage rate of antimicrobial agents for class I incision prevention was between 50% and 60%, as shown in the figure, and the use rate reduced dramatically when the medication proportion was restricted in October. Antimicrobial medicine usage declined in 2018 and 2019 compared to each month of 2017. The average usage rate in 2017 was 53.85 percent, while the use rate of antimicrobial drugs for class I incision prophylaxis was maintained between 35 and 50 percent in 2018 and 2019, reflecting a 10 percentage point decrease in the evaluation. Although current figures do not meet the national minimum of 30%, they have improved dramatically under the drug control system.

### 3.3. Top Ten Drugs by Amount of Medication

In 2017-2019, the top 10 drug goods by medication quantity were extremely varied (see Table 1). The top 10 in 2017 were all adjuvant medications, the top ten in 2018 contained two, and the rest were primarily therapeutic medications including antineoplastic drugs, anticoagulants, and anti-infective agents. Only one adjunct is in the top 10 in 2019, while the rest are both antineoplastic and antibacterial. Thus, it can be seen that the proportion of drugs took place through the implementation of control and control measures, the special management of adjuvant drugs, key monitoring drugs, and the promotion of physicians' awareness of rational drug use. Adjuvant drug use in hospitals has significantly decreased, with only one fifth of the number in 2018 from ten to one, and therapeutic drugs such as antitumor and antibacterial drugs account for eight, a significant proportion, in 2018.

### 3.4. Focus on Monitoring Drug Amounts

According to the most recent state key monitoring drug catalog for categorization data, see Figure 3 for a comparison of yearly medication usage in our hospital's key monitoring catalog from 2017 to 2019. As seen in the graph, the number of medications in each category declined in 2018 compared to 2017, and the reduction was greater. According to the statistics, the usage of concentrated monitoring declined by about 50% during the course of the year. 2019 is mostly unchanged from 2018.

## 4. Discussion

### 4.1. Exploration of the Effect of Drug Control System

Compared to 2017, the percentage of medications in 2018 and 2019 was all held at 30%, which fulfilled the criteria of national documents, via drug proportion control and control, antimicrobial drug administration, and key monitoring of drug administration [7]. The quantity of antimicrobial usage has fallen dramatically, and the rate of class I incision prophylactic antibiotic treatment has decreased by 10%, although not meeting national guidelines. Concentrated monitoring of the quantity of drug usage in the table of contents decreased by about 50%. The top 10 pharmaceuticals with the highest yearly drug usage quantities also changed structure; in 2017, they were all adjuvant drugs; in 2019, they were mostly antitumor, antibiotic, and other therapeutic drugs [8]. With the adoption of different regulations, numerous medical institutions around the nation began to regulate hospitals and obtained positive outcomes. Our control and control results show that the indicators meet or are close to the national requirements, but we recognize that the proportion of control drugs relates to various aspects of hospital clinical work, social relationship processing, and so on, and reflects the level of management work in the hospital function [9]. The functional department played an important management function in this control and control work, medical and technical departments provided a large amount of technical support, clinical departments with a positive attitude seriously summarized the deficiencies in the medication process and many aspects of the cooperation of multiple departments, so that the control and control work achieved better results [10]. Of course, the decreased drug ratio is undesirable for therapeutic purposes. The fundamental concerns of no indication medication, improper usage, and incorrect selection of antimicrobial kinds for perioperative prophylaxis are already evident in the prescription (medical claims) point review process, but additional minor issues continue to emerge in the point review results [11]. Currently, the drug ratio data has been maintained at about 30%; nevertheless, raising the degree of reasonable drug usage is our ultimate aim of ongoing drug management.

### 4.2. Focused Surveillance of Drugs and Medicare

The author compared the basic medical insurance, job injury insurance, and fertility insurance drug catalog of Hebei Province (2017 transition version) and the state-latest Medicare catalog of 2019, and two of the key monitored catalogs (gangliosides and bone peptides) were varieties that did not exist in either [12]. The original 2017 edition had four species (edaravone, alprostadil, murine nerve growth factor, and cinnarizide maleate), however, they were removed from the updated 2019 catalog [13]. The remaining 19 kinds were all novel category B medications introduced in Hebei Province in 2017. According to a notice issued by the state Medicare administration in 2019, each region must strictly enforce the drug catalog, not self-develop the catalog or increase the list of drugs with the method of transformation, and not self-adjust the set of restricted payment ranges for the drugs in the catalog. Stepwise digesting should take place over a three-year period for category B medications that are increased as specified in the initial provincial prescription list [14]. Provinces should preferentially modify out-of-pocket payments for medications that are included in the area of state focused surveillance during digestion. This means that by 2020, focused monitoring of varieties within the table of contents, six of which are not covered by Medicare and the other 19 newly added varieties, will be prioritized, implying that all varieties within the table of contents may not be in the Hebei Province Medicare table of contents. The continual decline in drug consumption in the table of contents is consistent with national policy, as represented in this drug control and control method. Then, in clinical practice, we provide medical services in accordance with national policy in order to be informed of changes in the Medicare catalog in a timely manner.

### 4.3. The Role of the Clinical Pharmacist in the Drug Control System

Clinical pharmacy has advanced rapidly in recent years, and clinical pharmacists at our hospital have contributed significantly to the drug control and control process [15]. Docking with clinical departments, each clinical pharmacist docks on professional departments to perform in-hospital medical order review on the responsible department, regularly announced the clinical department's morning meeting, pointed out deficiencies in the medication process, and provided advice to rationalize the medication [16]. Departments such as the combined medical department, laboratory, and hospital feeling carry out the rational drug use ward and walk into different clinical departments once a week. The clinical pharmacist was in charge of evaluating and discussing the department's medical recommendations in person. The requirements for perioperative prophylaxis and antimicrobial use in surgical departments, antimicrobial principles used in treatment, and adjunctive indications were all fully covered. It included in drug proportion control and control, antimicrobial drug double ranking, key monitoring of drug point review work, developing point review criteria, and monthly reporting of point review results to relevant functional departments in accordance with drug instructions and other strict controls. The reports focused on ongoing hospital-wide training, assessment, and timely interpretation of updated Medicare regulations, medication counseling for professionals, and so on.

## 5. Conclusion

In summary, all indicators such as the proportion of drugs in our hospital and the use rate of antimicrobial drugs for class I incision prevention have clearly improved under the current drug control and control system, the data meet the requirements at the same time, therapeutic drug use dominates, medication problems are improved, and medical staff awareness of rational drug use is increased. This implies that the intervention has a significant influence on the hospital drug control and control system, but it also improves physicians' rational drug use.

## Figures and Tables

**Figure 1:** The changes in the ratio of drug proportion from 2017 to 2019.

**Figure 2:** Utilization rate of prophylactic antibiotics for type I incisions from 2017 to 2019.

**Figure 3:** The amount of the key monitoring drugs from 2017 to 2019.

**Table 1:** The top ten drugs in the amount of medication from 2017 to 2019.

No.	2017	2018	2019
1	Lienal polypeptide injection	Imatinib mesylate	Meropenem
2	Creatine phosphate sodium for injection	Meropenem	Trastuzumab injection
3	Coenzyme complex	Sodium chloride 0.9%	Imatinib mesylate
4	Butylphthalide and sodium chloride injection	Cefoperazone tazobactam	Compound porcine cerebroside and ganglioside injection
5	Edaravone	Lienal polypeptide injection	Cefoperazone tazobactam
6	Calf spleen extract	Cefazolin sodium	Cefamandole
7	Lansoprazole needle	Sodium chloride 0.9% (double valve soft bag)	Paclitaxel liposome for injection
8	Placental polypeptide injection	Ginkgolide injection	Piperacillin sodium and tazobactam sodium
9	Omeprazole	Nadroparin calcium	Cefazolin
10	Brain glycoside carnosine	Piperacillin sodium and tazobactam sodium	Sodium chloride 0.9% (double pipe and double plug)

## Data Availability

All of the data in this article is actually available within the article.
